# Bayesian Fully Convolutional Networks for Brain Image Registration

**DOI:** 10.1155/2021/5528160

**Published:** 2021-07-26

**Authors:** Kunpeng Cui, Panpan Fu, Yinghao Li, Yusong Lin

**Affiliations:** ^1^School of Information Engineering, Zhengzhou University, Zhengzhou 450001, Henan, China; ^2^Collaborative Innovation Center for Internet Healthcare, Zhengzhou University, Zhengzhou 450052, Henan, China; ^3^School of Software, Zhengzhou University, Zhengzhou 450002, Henan, China; ^4^Hanwei IoT Institute, Zhengzhou University, Zhengzhou 450002, Henan, China

## Abstract

The purpose of medical image registration is to find geometric transformations that align two medical images so that the corresponding voxels on two images are spatially consistent. Nonrigid medical image registration is a key step in medical image processing, such as image comparison, data fusion, target recognition, and pathological change analysis. Existing registration methods only consider registration accuracy but largely neglect the uncertainty of registration results. In this work, a method based on the Bayesian fully convolutional neural network is proposed for nonrigid medical image registration. The proposed method can generate a geometric uncertainty map to calculate the uncertainty of registration results. This uncertainty can be interpreted as a confidence interval, which is essential for judging whether the source data are abnormal. Moreover, the proposed method introduces group normalization, which is conducive to the network convergence of the Bayesian neural network. Some representative learning-based image registration methods are compared with the proposed method on different image datasets. Experimental results show that the registration accuracy of the proposed method is better than that of the methods, and its antifolding performance is comparable to that of fast image registration and VoxelMorph. Furthermore, the proposed method can evaluate the uncertainty of registration results.

## 1. Introduction

Image registration is an image-processing process that aligns two or more images of the same scene captured at different times and different perspectives or by using different sensors [1, 2]. Nonrigid medical image registration is a key step in medical image processing. In clinical diagnosis, it can judge a patient's progress by aligning the brain magnetic resonance images of the patient with Alzheimer's disease at different periods [3, 4]. In tumor surgery, rapid medical image registration can aid doctors in surgical navigation [5–7]. In demography research, image registration is helpful for studying differences in the brain tissue structures of people from different countries.

With the advances in medical image registration technology, various registration methods have been developed, such as elastic body models [8–10], viscous fluid flow models [11–13], diffusion models [14], curvature registration [15], statistical parameter mapping [16], free-form deformation with b-spline [17], discrete method [18, 19], and demons [20] for registration model construction. Many optimization algorithms have also been devised, such as gradient descent methods [21], conjugate gradient methods [22, 23], Powell's conjugate direction method [24, 25], quasi-Newton methods [26, 27], Gauss–Newton method [28, 29], and stochastic gradient descent methods [30, 31]. Similarity measurement methods, such as the sum of squared differences [32], the sum of absolute differences, cross-correlation [33], and mutual information [34], have been proposed.

However, traditional registration methods face real-time challenges. Large amounts of input data must be processed when performing nonrigid registration modeling on 3D data with high resolution, a step that requires a long time. The optimization part usually uses an iterative algorithm, thereby further increasing the total time needed to obtain the final result [35].

With the development of deep learning, several researchers have proposed deep neural networks to learn features of unregistered images. Registration methods based on deep learning can be supervised [36, 37] or unsupervised [38–40]. Most supervised registration methods rely on anatomical labels. However, marking anatomical labels is difficult, a step that not only consumes a lot of time of experts but also sometimes hardly guarantees accuracy. In practice, supervised registration methods are restricted. In their place, some scholars have proposed unsupervised medical image registration methods.

Several unsupervised medical image registration methods have been proposed. VoxelMorph, a recently proposed unsupervised learning-based method for deformable medical image registration, has a better registration accuracy and a faster speed than other registration methods [41]. Some researchers combined the advantages of classical methods and learning-based methods to produce a probabilistic generative model and derive a diffeomorphic inference algorithm [42]. A registration method called fast image registration (FAIM) for 3D medical image registration has been proposed. Compared with the registration network based on U-net, FAIM has fewer trainable parameters to obtain a higher registration accuracy. In addition, FAIM has less irreversible regions because of the penalty loss for negative Jacobian determinants [43]. Some scholars recently proposed the Probab-Mul registration method, which is a feature-level probability model that can perform regularization on the hidden layers of two deep convolutional neural networks [44].

The focus of the present study is mainly on the accuracy of registration methods and barely on the uncertainty of their registration results. The uncertainty of registration results is very important in clinical applications as it can be used to judge whether the registration result is meaningful. For example, if a model is modeling normal human brain images, it will never see abnormal brain images that have brain tumors, malformations, and edema. When the uncertainty of a registration result is higher than a certain threshold, the source image can be judged as an abnormal brain image. During testing, the Bayesian neural network can obtain the uncertainty of results. Bayesian neural networks are used in autonomous driving, classification tasks, and segmentation tasks. Some researchers recently applied Bayesian neural networks to image registration. Deshpande et al. employed a Bayesian deep learning approach for deformable medical image registration. They reported that this approach has a better performance than existing state-of-the-art approaches [45]. Khawaled et al. developed a fully Bayesian framework for unsupervised deep learning-based deformable image registration. Their approach provided better estimates of the deformation field, thereby improving registration accuracy [46]. However, these aforementioned methods do not sufficiently consider and discuss the uncertainty of registration results. Furthermore, they are suitable for 2D images only.

In this paper, a method based on Bayesian fully convolutional networks is proposed for image registration. The proposed method generates a geometric uncertainty map to measure the uncertainty of registration results. Thus, when the source image obtained is abnormal data, the model will provide a hint that the source image is problematic instead of immediately accepting the registration result of the model. Group normalization (GN) is also added in networks. GN groups channel similar features into one group. Hence, GN can make the model easier to optimize and converge to improve registration accuracy. The performance of the registration model in evaluating uncertainty is determined.

This paper is organized as follows.  Section 2 introduces the principle of the proposed method.  Section 3 describes the experimental setup.  Section 4 discusses the experimental results. Finally, Section 5 summarizes the results of the study and considers directions for future work.

## 2. Methods

Figure 1 presents an overview of the proposed method. We used CNN to model the function *g*_*γ*_(*S*, *T*) = *u*, where *γ* is the parameter of the convolutional layers, *S* is the source image, *T* is the target image, and *u* is the displacement field between the source image and the target image. *S* and *T* are defined over a 3D spatial domain Ω ⊂ *R*^3^. For each voxel *p* ∈ Ω, *u*(*p*) is the displacement, where the map *ϕ*=*Id*+*u* is formed using an identity transform and *u*. The network takes *S* and *T* as the input and uses a set of parameters *γ* to calculate *ϕ*. We used a spatial transformation function to warp *S* to *S*∘*ϕ* and evaluate the similarity between S∘*ϕ* and *T*. During testing, given the images *T* and *S* of the test set, we obtained the registration field by evaluating *g*_*γ*_(*S*, *T*).

### 2.1. Architecture

In this section, the architecture of the convolutional neural network used in the proposed method is described in detail (Figure 2). During training, the moving image and the target image are stacked together as the input fed into the Bayesian fully convolutional network module (BFCNM) [43]. The first layer is inspired by Google's inception module. The purpose of this layer is to compare and capture information on different spatial scales of later registration. Parametric rectified linear unit [47] activation is utilized at the end of each convolution block, and linear activation is employed in the last layer to generate the displacement field. Instead of inserting max-pooling layers, a kernel stride of 2 is used to reduce image size. Three “add” skip connections are present in downsampling and upsampling [43]. The “add” skip connection is conducive to the fusion of upsampling information and its corresponding downsampling information. During the upsampling phase, two Bayesian blocks are used. The Bayesian blocks are composed of a transposed convolutional layer, a convolutional layer, PReLU, a group normalization layer, and a Dropout layer. The detail of the Bayesian block is shown in Figure 2(b). In this paper, Monte Carlo Dropout (MC-Dropout) is introduced; it is interpreted as a Bayesian approximation of Gaussian processes.

### 2.2. Spatial Transformation Function

The spatial transformation function uses the *ϕ* generated by BFCNM to resample *S* and obtain the warped image *S*∘*ϕ*. The proposed method learns the optimal parameter values by minimizing the difference between *S*∘*ϕ* and *T*. A differentiable operation is constructed on the basis of the spatial transformer network [41, 48] via the standard gradient-based method to calculate *S*∘*ϕ*. For each voxel *p*, a voxel position *p*′ = *p* + *u*(*p*) is calculated in the source image. The image values are only defined in integer positions. Thus, linear interpolation is performed at eight adjacent voxels:

(1) $$\begin{array}{c} S\circ \phi \left(p\right)=\sum_{q\in Z\left(p^{\prime }\right)}S\left(q\right)\prod_{d\in \left\{x,y,z\right\}}\left(1-\left|p_{d}^{\prime }-q_{d}\right|\right). \end{array}$$

where *Z*(*p*′) is the voxel neighbors of *p*′ and *d* is iterated in the dimension of Ω. Errors can be backpropagated during the optimization process because gradients or subgradients can be calculated.

### 2.3. Loss Function

The total training loss is the sum of an image dissimilarity term *L*_image_ and the regularization terms, as shown in Table 1. The loss function [43] is defined as follows:

(2) $$\begin{array}{c} L_{\text{total}}=L_{\text{image}}\left(S,T\right)+\alpha R_{1}\left(u\right)+\beta R_{2}\left(u\right). \end{array}$$

The main loss *L*_image_ with cross-correlation (CC) in this paper is for the similarity between the warped source image and the target image. The definition of CC is as follows:

(3) $$\begin{array}{c} \text{CC}\left(t,s\circ \phi \right)=\frac{{\left(\sum_{x\in \Omega }\left(t\left(x\right)-\bar{t}\left(x\right)\right)\left(s\circ \phi \left(x\right)-\bar{s\circ \phi }\left(x\right)\right)\right)}^{2}}{\left(\sum_{x\in \Omega }{\left(t\left(x\right)-\bar{t}\left(x\right)\right)}^{2}\right)\left(\sum_{x\in \Omega }{\left(s\circ \phi \left(x\right)-\bar{s\circ \phi }\left(x\right)\right)}^{2}\right)}, \end{array}$$

where *t*(*x*) is the grey value of the target image, $\bar{t}\left(x\right)$ is the average grey value of the target image, *s*∘*ϕ*(*x*) is the grey value of the warped image, and $\bar{s\circ \phi }\left(x\right)$ is the average grey value of the warped image.

The first regularization term *R*_1_ regularizes the overall smoothness of the predicted displacements. The parameter of the regular term is *α*, and its value is always 1. The purpose of the second regularization is to penalize transformations that have many negative Jacobian determinants. The parameter of the regular term is *β*. The transformations of all nonnegative Jacobian determinants will not be penalized. If the Jacobian determinant is negative, then the transformation result will be folded, which is physically unrealistic.

### 2.4. Group Normalization

Group normalization (GN) is a feature-normalization technique that is inserted into the architecture of deep neural networks as a trainable process. The purpose of GN is to reduce internal covariant shifts. With training iterations, the distribution of features often continuously changes. Under this condition, the parameters in the convolutional layer must be continuously updated to adapt to the changes in distribution. GN normalizes the feature to a fixed distribution (mean value is zero, and the standard deviation is 1) and then adjusts the feature to an ideal distribution, which is learned in the training process [48].

Here, *x* is the feature computed by a layer, and *i* is an index. In the case of 3D images, *i*=(*i*_*N*_, *i*_*C*_, *i*_*D*_, *i*_*H*_, *i*_*W*_) is a 5D vector indexing the features in (*N*, *C*, *D*, *H*, *W*) order, where *N* is the batch axis; *C* is the channel axis; and *D*, *H*, and *W* are the spatial depth, height, and width axes, respectively.

Formally, the group normalization layer must compute for mean *µ* and standard deviation *σ* in a set *S*_*i*_. *S*_*i*_ is a group and defined as follows:

(4) $$\begin{array}{c} S_{i}=\left\{k|k_{N}=i_{N},\left\lfloor \frac{k_{C}}{C/G}\right\rfloor =\left\lfloor \frac{i_{C}}{C/G}\right\rfloor \right\}, \end{array}$$

where *G* is the number of groups, which is a predefined hyperparameter; *C*/*G* is the number of channels in each group; ⌊·⌋ represents floor operation; ⌊*k*_*C*_/(*C*/*G*)⌋=⌊*i*_*C*_/(*C*/*G*)⌋ means that the indexes *i* and *k* are in the same group of channels, assuming that each group of channels is stored in sequential order along the *C* axis; and *S*_*i*_ contains all voxels along the (*D*, *H*, *W*) axes and along with a group of (*C*/*G*) channels.

The mean *μ*_*i*_ and standard deviation *σ*_*i*_ of *S*_*i*_ are computed as follows:

(5) $$\begin{array}{c} \mu_{i}=\frac{1}{m}\sum_{k\in S_{i}}x_{k},\\ \sigma_{i}=\sqrt{\frac{1}{m}\sum_{k\in S_{i}}{\left(x_{k}-\mu_{i}\right)}^{2}+\varepsilon }, \end{array}$$

where *ε* is a small constant, and *m* is the size of set *S*_*i*_. GN then performs the following computation:

(6) $$\begin{array}{c} {\hat{x}}_{i}=\frac{1}{\sigma_{i}}\left(x_{i}-\mu_{i}\right), \end{array}$$

GN learns a per-channel linear transform to compensate for the possible loss of representational ability:

(7) $$\begin{array}{c} y_{i}=\gamma {\hat{x}}_{i}+\beta , \end{array}$$

where *γ* and *β* are trainable scale and shift, respectively. Given the *S*_*i*_ in (4), the GN layer is defined by equations (5)–(7). Specifically, the voxels in the same group are normalized by the same *μ*_*i*_ and *σ*_*i*_. GN also learns the *γ* and *β* of each channel.

### 2.5. Bayesian Neural Network

In this section, the registration network based on Bayesian inference is introduced. The credibility of the results is important in solving medical problems. Several researchers proposed a Bayesian neural network by studying the uncertainty of deep learning [49, 50]. The Bayesian neural network is a statistical model derived from the perspective of probability. The parameters in the model are initialized by an a priori distribution, and the parameters are further optimized by Bayesian inference. In the Bayesian neural network, given the data set *D* and weight *W*, the dataset *D* contains data *X* and label *Y*. The goal of Bayesian neural network training is to optimize the parameters, that is, to seek the posterior distribution of weight *W*. According to Bayesian criterion, the posterior distribution of weight *W* is written as

(8) $$\begin{array}{c} p\left(W|D\right)=\frac{p\left(D|W\right)p\left(W\right)}{p\left(D\right)}\\ =\frac{p\left(y|x,W\right)p\left(W\right)}{p\left(y|x\right)}, \end{array}$$

where *x* and *y* are the data in the training set and the corresponding label, respectively, and *p*(*W*) is the initial value of the parameter (i.e., the prior distribution). The posterior distribution of the labels predicted by the Bayesian neural network can then be calculated as follows [51]:

(9) $$\begin{array}{c} p\left(y^{*}|x^{*},D\right)=E_{p\left(W|D\right)}\left[p\left(y^{*}|x^{*},W\right)\right]=\int p\left(y^{*}|x^{*},W\right)p\left(W|D\right)dW. \end{array}$$

In equation (9), the weight parameter *W* in the network is used to predict the unknown distribution of label *y*^*∗*^. In the Bayesian neural network model, the solution of the posterior distribution *p*(*W|D*) of the parameters is the key to the entire model. However, this solution is computationally intractable for neural networks of any size. Therefore, many researchers use approximate methods to obtain the solution [52, 53].

A common approach is to use variational inference to approximate the posterior distribution of the weights. This method introduces the variational distribution *q*_*θ*_(*W*) of weight *w*, which is parameterized on *θ*. The approximate posterior distribution *q*_*θ*_(*W*) is obtained by minimizing the Kullback-Leibler (KL) divergence between *q*_*θ*_(*W*) and the true posterior distribution *p*(*W|D*).

(10) $$\begin{array}{c} \mathrm{KL}\left(\left.q_{\theta }\left(W\right)\right\|p\left(W|D\right)\right). \end{array}$$

Minimizing KL divergence is equivalent to minimizing the Negative Evidence Lower Bound (NELBO):

(11) $$\begin{array}{c} \mathrm{NELBO}=E_{q_{\theta }}\left[-\log\;p\left(Y|X,W\right)\right]\\ +\mathrm{KL}\left(\left.q_{\theta }\left(W\right)\right\|p\left(W\right)\right)\\ =-\int q_{\theta }\left(W\right)\log\;p\left(Y|X,W\right)dW\\ +\mathrm{KL}\left(\left.q_{\theta }\left(W\right)\right\|p\left(W\right)\right), \end{array}$$

with respect to the variational parameter *θ*. The first term (commonly referred to as the expected log-likelihood) encourages *q*_*θ*_(*W*) to place its mass on the configurations of the latent variable that explains the observed data. However, the second term (referred to as prior KL) encourages *q*_*θ*_(*W*) to be similar to the prior distribution *p*(*W*), preventing the model from overfitting. The goal is to develop an explicit and accurate approximation for the expectation.

Our approach uses Bernoulli approximating variational inference and Monte Carlo sampling [54]. In practice, Dropout is used for Bayesian neural network approximation.

When Dropout [55] is applied to the output of a layer, the output can be written as

(12) $$\begin{array}{c} a_{i}^{\text{DO}}=\sigma \left(z_{i}⊙\left(W_{i}v\right)\right). \end{array}$$

where, for a single *K*_*i*−1_ dimensional input *v*, the *i*^th^ layer of a neural network with *K*_*i*_ units would output a *K*_*i*_ dimensional activation vector; *w*_*i*_ is the *K*_*i*_ × *K*_*i*−1_ weight matrix; *σ*(·) is the nonlinear activation function; ⊙ signifies the Hadamard product; *z*_*i*_ is a *K*_*i*_ dimensional binary vector with its elements drawn independently from *z*_*i*_^(*k*)^ ~ Bernoulli(*p*_*i*_)*k* = 1,…, *K*_*i*_; and *p*_*i*_ is the probability of keeping the output activation.

The solution of the posterior distribution *p*(*W|D*) of the parameters is further improved after introducing the Bernoulli distribution into the weight parameters of our model. The Monte Carlo sampling method is used to estimate the first item in (11):

(13) $$\begin{array}{c} E_{q_{\theta }}\log\;p\left(Y|X,W\right)=\sum_{n=1}^{N}\int q_{\theta }\left(W\right)\log\;p\left(y_{n}|x_{n},W\right)\\ =\frac{1}{N}\sum_{n=1}^{N}\log\;p\left(y_{n}|x_{n},{\hat{W}}_{n}\right), \end{array}$$

where ${\overset{\wedge }{W}}_{n}$ is not the maximum posterior estimation but the random variable realizations from the Bernoulli distribution; and ${\overset{\wedge }{W}}_{n}∼q_{\theta }\left(W\right)$, which is the same as applying Dropout to the weights of the network. For the second item in equation (11) (i.e., KL term), the approximate solution is given in the literature [56]. The KL term has been shown to be equivalent to ∑_*i*=1_^*L*^‖*W*_*i*_‖_2_^2^. Thus, equation (11) can be rewritten as

(14) $$\begin{array}{c} \mathrm{NELBO}=-\frac{1}{N}\sum_{n=1}^{N}\log\;p\left(y_{n}|x_{n},{\hat{W}}_{n}\right)+\sum_{i=1}^{L}{\left\|W_{i}\right\|}_{2}^{2}. \end{array}$$

Equation (14) is the unbiased estimation of equation (11). Interestingly, it is the same as the loss function used in standard neural networks with *L*_2_ weight regularization, and Dropout is applied to all weights of the network. Therefore, training such a neural network with stochastic gradient descent has the same effect as minimizing the KL term in (10). This scheme is similar to a Bayesian neural network and can generate a set of parameters that can best explain the observed data while preventing overfitting.

Predictions in this model follow (9) replacing the posterior *p*(*W|D*) with the approximate posterior *q*_*θ*_(*W*). The integral can be approximated with Monte Carlo integration [51, 54]:

(15) $$\begin{array}{c} p\left(y^{*}|x^{*},D\right)\approx \int p\left(y^{*}|x^{*},W\right)q_{\theta }\left(W\right)\text{d}W\\ \approx \frac{1}{T}\sum_{t=1}^{T}\log\;p\left(y_{n}|x_{n},{\hat{W}}_{t}\right)\\ \approx p_{MC}\left(y^{*}|x^{*}\right), \end{array}$$

where ${\overset{\wedge }{W}}_{t}∼q_{\theta }\left(W\right)$, which means that, at test time, the Dropout layers are kept active to keep the Bernoulli distribution over the network weights. This integration is referred to as the Monte Carlo Dropout.

The Monte Carlo Dropout reflects the need to conduct multiple forward propagation processes on the same input. In this manner, the output of “different network structures” can be obtained under the action of Dropout during testing. The prediction results and the uncertainty of the model can be obtained by calculating the average and statistical variance of these outputs. The advantage of Bayesian deep learning is that Monte Carlo Dropout can give a prediction value and the confidence of the predicted value.

### 2.6. Measuring Model Uncertainty

Uncertainties in a network are a measure of how certain the model is with its prediction. In general, Bayesian modeling has two types of uncertainty. Model uncertainty, also known as Epistemic uncertainty, measures what the model does not know owing to the lack of training data. This uncertainty can be reduced with more data. During testing, model uncertainty can measure whether the testing data exists in the distribution of the training data. Aleatoric uncertainty measures the noise inherent in the observation data and cannot be reduced by collecting more data [51].

By computing the result of stochastic forward passes of the Bayesian neural network, the model's confidence of its output can be estimated. In this paper, the mean *μ* and the standard deviation *σ* of all displacements produced by Monte Carlo sampling are calculated. The mean *μ* is used in the registration image, whereas the standard deviation *σ* provides an estimate of the uncertainty of registration results. The mean *μ* of the displacement fields is calculated as follows:

(16) $$\begin{array}{c} \mu =\frac{1}{M}\sum_{i=1}^{M}y_{i}, \end{array}$$

where *M* represents the number of Monte Carlo sampling (*M* = 48 in this paper). *y*_*i*_ represents the displacement field sampled by *i*th. After calculating the mean value of the displacement fields, the standard variance of the displacement fields can be calculated as follows:

(17) $$\begin{array}{c} \sigma =\sqrt{\frac{1}{M-1}\sum_{i=1}^{M}{\left(y_{i}-\mu \right)}^{2}}, \end{array}$$

where *σ* can be expressed as the uncertainty of registration results.

## 3. Experiment

### 3.1. Experimental Setup

The dataset we adopted herein was created by Arno et al. who based it on a collection of 101 T1-weighted MRIs from healthy subjects [57]. In this paper, we used brain images from the four subsets of Mindboggle101, namely, NKI-RS-22, NKI-TRT-20, MMRR-21, and OASIS-TRT-20, for a total of 83 images. These images are already warped to MNI152 space. Each image had a dimension of 182 × 218 × 182, each of which we truncated to 144 × 180 × 144. In the preprocessing stage, we utilized the FMRIB Software Library (FSL) to perform affine registration on NKI-RS-22, NKI-TRT-20, MMRR-21, and OASIS-TRT-20. We initially normalized the voxel intensity of each brain image and then normalized voxel intensity to 0–255. Finally, we performed a registration test on the five main anatomical regions of the cerebral cortex.

### 3.2. Evaluation Metrics

#### 3.2.1. Dice Scores

If the registration field *ϕ* represents an accurate correspondence, then the corresponding anatomical regions in *T* and S∘*ϕ* should overlap well. Therefore, we evaluated registration accuracy by using the Dice score. The Dice score is defined as follows [43]:

(18) $$\begin{array}{c} \mathrm{DICE}=\frac{2*\left|X\cap Y\right|}{\left|X\right|+\left|Y\right|}. \end{array}$$

#### 3.2.2. Regularized Penalty Folding

We also evaluated the regularity of deformation fields. Specifically, the Jacobian matrix captures the local properties of *ϕ* around voxel *p*. We counted all nonbackground voxels where the Jacobian determinant det(∇*ϕ*) < 0 is negative [43]:

(19) $$\begin{array}{c} N≔\sum \delta \left(\det\left(D\phi \right)<0\right), \end{array}$$

where *δ*(·) indicates that if it is true, then the return value is 1.

#### 3.2.3. Uncertainty Evaluation Metrics

We adopted the method proposed in the literature to evaluate uncertainty performance [51]. We used metrics that incorporate the ground truth label, model prediction, and uncertainty value to evaluate the performance of such models in estimating uncertainty.  Figure 3 shows the required processing steps to prepare these quantities for our metrics in a registration example. We computed the map of correct and incorrect values by matching the ground truth labels and the model predictions. We converted the uncertainty map into a map of certain and uncertain predictions by setting the uncertainty threshold *T*, which varies between the minimum and the maximum uncertainty values in the entire test set. The following indicators can reflect the characteristics of a good uncertainty estimator.

Negative predictive value (NPV): in the output of certain results by the model, NPV is the percentage of voxels that is correctly predicted and can be written as a conditional probability:

(20) $$\begin{array}{c} \mathrm{NPV}=\frac{P\left(\mathrm{correct},\mathrm{certain}\right)}{P\left(\mathrm{certain}\right)}=\frac{\mathrm{TN}}{\mathrm{TN}+\mathrm{FN}}. \end{array}$$

True positive rate (TPR): if a model is making an incorrect prediction, then the proportion of uncertain voxels is called TPR. TPR can be written as a conditional probability:

(21) $$\begin{array}{c} \mathrm{TPR}=\frac{P\left(\mathrm{uncertain},\mathrm{incorrect}\right)}{P\left(\mathrm{incorrect}\right)}=\frac{\mathrm{TP}}{\mathrm{TP}+\mathrm{FN}}. \end{array}$$

Uncertainty accuracy (UA): UA is the overall accuracy of uncertainty estimation and can be measured as the ratio of the desired cases explained above (TP and TN) over all possible cases:

(22) $$\begin{array}{c} \mathrm{UA}=\frac{P\left(\mathrm{correct},\mathrm{certain}\right)+P\left(\mathrm{uncertain},\mathrm{incorrect}\right)}{P\left(\mathrm{correct}\right)+P\left(\mathrm{incorrect}\right)}=\frac{\mathrm{TP+TN}}{\mathrm{TP+TN+FP+FN}}. \end{array}$$

Clearly, in all the metrics proposed above, higher values indicate that the model performs better. The values of these metrics depend on the uncertainty threshold.

### 3.3. Baseline Methods

In the comparative study, we used FSL, a comprehensive library of analytical tools for fMRI, MRI, and diffusion tensor imaging brain imaging data, as the baseline to perform an affine registration experiment with 12 degrees of freedom on the test set. We used the second baseline symmetric normalization (SyN) with mutual information as a similarity measure in the publicly available Advanced Normalization Tools (ANTs) software package [58]. We also tested the recently developed CNN-based methods, namely, VoxelMorph [41], FAIM [43], and Probab-Mul [44], and compared their performance with that of the proposed method. The hyperparameters of the CNN-based methods were consistent. Finally, we adopted various methods for ablation study. The method that only adds GN was denoted as Our-GN, and the method that only adds Dropout was labeled as Our-DO. These two methods were consistent with our method in terms of hyperparameter settings.

### 3.4. Implementation

We divided the data set into training and test image sets. The training set consisted of all ordered brain image pairs from the union of the NKI-RS-22, NKI-TRT-20, and MMRR-21 subsets, which comprised 3906 pairs in total. The test set consisted of all ordered pairs from the OASIS-TRT-20 subset with 380 pairs in total. We trained FAIM, VoxelMorph, Probab-Mul, and our method on all pairs of images from the training set and then examined their predicted deformations by using the pairs of images from the testing set.

We implemented our method using Keras [59] with a Tensorflow backend [60]. We used the Adam optimizer. We trained three networks with the same hyperparameters: batch size = 1, learning rate = 10^−4^, epochs = 10, and *α* = 1.

## 4. Results and Discussion

In this experiment, we separately trained the proposed networks with different *β* values. We optimized the parameters by the validation set and reported results in our test set. The predicted deformation field could not guarantee diffeomorphism; therefore, the transformation of irreversible regions caused an image to “fold” on itself. In these regions, the determinant of the Jacobian matrix of the deformation field was negative (Figure 4). However, spatial folding is physically impossible; hence, this phenomenon causes registration errors in clinical applications. The frequency of such errors limits the application of neural networks in image registration.

### 4.1. Dice Scores

The mean Dice scores of the different methods across all predicted labels with their corresponding target labels are shown in Table 2. We selected five scales of regularization strength *β* from 0 to 10^−2^. Results showed that FSL was not suitable for fine registration because of its few registration parameters in the affine registration with 12 degrees of freedom. ANT (SyN) is a nonrigid registration method, and its registration accuracy was found to be higher than that of affine registration. The Dice scores of FAIM slightly decreased as *β* increased, and its Dice scores were higher than those of VoxelMorph. The registration accuracy of Probab-Mul was slightly better than that of FAIM. The proposed method achieved the highest registration accuracy under all *β* values.

The results of the ablation study revealed that the Dice score of Our-GN was higher than FAIM by 2.8% on average (Table 2). Experimental results showed that GN could improve the accuracy of registration. Moreover, the registration accuracy of Our-DO was slightly lower than that of FAIM (Table 2), illustrating that adding a Dropout layer had little impact on registration accuracy.

When *β* takes 0,  10^−5^, 10^−4^10^−3^, and 10^−2^, the Dice scores of our method were higher than those of FAIM by 2.63%, 2.80%, 2.84%, 2.50%, and 3.37%, respectively, higher than those of Probab-Mul by 2.31%, 2.49%, 2.55%, 2.05%, and 2.88%, respectively, and higher than those of VoxelMorph by 4.78%, 5.17%, 5.27%, 5.21%, and 5.90%, respectively (Table 2). This result implied that inserting GN layers into the network architecture could indeed enable the network to learn better parameters and could make the network easier to optimize and converge, thereby improving registration accuracy. During training, we set epochs = 10, and each epoch took about 100 min to perform 2900 iterations.

Figure 5 presents the boxplot of the Dice scores of the five main anatomical regions of the cerebral cortex when *β* = 10^−3^. The Dice scores of ANTs in each label were quite different, indicating that ANTs were unstable. The flatness of the boxplots indicated that the stability of the proposed method was comparable to that of other deep learning methods. The proposed method achieved the highest registration accuracy in the five regions of the cerebral cortex.

Figure 6 shows the mean Dice scores corresponding to the different *β* values of all methods. The accuracy of the proposed method was relatively consistent with different *β* values and was higher than that of the other methods.

### 4.2. Data-Regularized Penalty Folding

Figure 7 visualizes the effects of the second regularization term *R*_2_ (*u*), which directly penalized “foldings” during training. *β* = 0 means the regularization was not used, and multiple locations were visible in the transformation whose Jacobian determinants were negative. The number of “foldings” voxels greatly reduced when *β* = 10^−5^. Only several “folding” voxels were observed when *β* = 10^−4^. The number of “folding” voxels was almost eliminated when *β* = 10^−3^.

We listed the mean values of the number of voxels of different methods whose Jacobian determinants were negative in Table 3. The proposed method had a lower number of “foldings” in the predicted deformations as *β* increased.

### 4.3. Uncertainty Measure

In this section, the performance of the registration model in estimating uncertainty was evaluated.  Figure 8 shows the results of uncertainty evaluation by the proposed method. In the experiment, the Dropout rate of the Dropout layer was set to 0.5. During the test, the Dropout layer was always on, and 48 Monte Carlo samplings were performed. The threshold *T* of the uncertainty map had an impact on the uncertainty measure. We set the threshold between 0 and 1 with an interval of 0.1. As the threshold increased, the proportion of the uncertain part of the uncertainty map decreased; hence, the TPR curve gradually decreased. The maximum value of 0.756 in the NPV measurement was obtained at the threshold of 0.1. This value slightly decreased as the threshold further increased but still greater than 0.72. If the model was certain about its prediction, then the accuracy of the prediction was higher. Uncertainty accuracy was also the largest (0.77) when the threshold was 0.1 and slightly declined as the threshold further increased. It remained greater than 0.712. Uncertainty accuracy is the overall accuracy of uncertainty measurements. It shows the ratio of the cases we desired in all possible cases. The uncertainty accuracy of our model was relatively high (Figure 8).

## 5. Conclusion

We developed an unsupervised 3D medical image registration method that uses Bayesian fully convolutional networks for registration. The proposed method introduces probability distributions for network weights and obtains the uncertainty of registration results. We introduced GN into the neural network architecture, which is conducive to the optimization and convergence of the neural network. The experimental results showed that the proposed method can obtain higher registration Dice scores than other state-of-the-art models and achieve an antifolding performance comparable to that of FAIM and VoxelMorph. The proposed method can also estimate the uncertainty of registration results. Although penalty folding can reduce the irreversible area of registration result, it cannot guarantee that the irreversible area is zero. Thus, the nonrigid registration of diffeomorphism with high accuracy is one of our research directions in the future.

## Figures and Tables

**Figure 1:** Overview of the method.

**Figure 2:** Convolution network architecture implementing BFCNM (*g*_*γ*_(*S*, *T*)). (a) Highest-level view, showing sequential Conv3D and Bayesian block. (b) Details of Bayesian block.

**Figure 3:** Overview of the metrics for the evaluation of the uncertainty quality in a registration example.

**Figure 4:** The first and last images are the source and target images, respectively, and the third image is the deformed image produced by the method. The second image shows the values of the Jacobian determinant of the predicted deformation with “folding” locations (negative determinant) marked in red. The deformed grids illustrate parts of the deformation. (a) Source, (b) deformation, (c) deformed, and (d) target.

**Figure 5:** Boxplots of Dice scores for five main anatomical structures of the cerebral cortex.

**Figure 6:** Mean Dice score corresponding to the different *β* of all methods.

**Figure 7:** Locations where det(∇*ϕ*) < 0 (marked in dark blue) with different *β* shown on one slice. Predictions were done using the proposed method. (a) 0, (b) *β* = 10^−5^, (c) *β* = 10^−4^, and (d) *β* = 10^−3^.

**Figure 8:** Quantitative uncertainty estimation performance for registration task using the evaluation metrics. The abscissa is the threshold (*T*). The ordinate is negative predictive value (NPV), true positive rate (TPR), and uncertainty accuracy (UA), respectively.

**Table 1:** Loss and regularization functions used.

*L*_image_(*S*, *T*): 1 − CC(*S*∘*ϕ*^−1^, *T*)
Regularization: *R*_1_(*u*)=‖*Du*‖_2_
Regularization: *R*_2_(*u*)=0.5(|det(*Dϕ*^−1^)| − det(*Dϕ*^−1^))

**Table 2:** Mean Dice scores with different *β* values.

Mean Dice	*β* = 0	*β* = 10^−5^	*β* = 10^−4^	*β* = 10^−3^	*β*=10^−2^
FSL (Affine)	0.4357	—	—	—	—
ANTs(SyN)	0.5139	—	—	—	—
VoxelMorph	0.5255	0.5203	0.5165	0.5091	0.4908
FAIM	0.5470	0.5440	0.5408	0.5362	0.5161
Probab-Mul	0.5502	0.5471	0.5437	0.5407	0.5210
Our-DO	0.5459	0.5421	0.5380	0.5323	0.5149
Our-GN	0.5729	0.5709	0.5679	0.5591	0.5410
Our method	**0.5733**	**0.5720**	**0.5692**	**0.5612**	**0.5498**

Bold values mean the optimal dice score of all methods at the same *β* value.

**Table 3:** Mean number of “folding” locations with different *β* values.

Mean *N*	*β* = 0	*β* = 10^−5^	*β* = 10^−4^	*β* = 10^−3^	*β* = 10^−2^
VoxelMorph	33733	1400	232	60	13
FAIM	39377	1531	234	26	3
Probab-Mul	39905	1700	241	28	6
Our method	39842	1680	240	25	3

## Data Availability

All datasets used to support the findings of this study were supplied by the publicly available Mindboggle101 database. The URL to access this data is https://osf.io/yhkde/.
